The article "Recognition of Continuous Music Segments Based on the Phase Space Reconstruction Method" was retracted in 2023. Reasons: unreliable results or conclusions; concerns about the data; concerns about the peer review; concerns about the citations.

# Recognition of Continuous Music Segments Based on the Phase Space Reconstruction Method

**DOI:** 10.1155/2022/4099505

**Published:** 2022-10-04

**Authors:** Xuesheng Huang, YanQing Hu

**Affiliations:** ^1^School of Music and Dance, Quanzhou Normal University, Quanzhou, Fujian 362000, China; ^2^Dean's Office, Quanzhou Normal University, Quanzhou, Fujian 362000, China

## Abstract

Piano score recognition is one of the important research contents in the field of music information retrieval, and it plays an important role in information processing. In order to reduce the influence of vocals on the progress of piano notes and restore the harmonic information corresponding to piano notes, the article models the harmonic information and vocal information corresponding to piano notes in the frequency spectrum. We use the phase space reconstruction method to extract the nonlinear feature parameters in the note audio and use some of the parameters as the training set to construct the support vector machine (SVM) classifier and the other part as the test set to test the recognition effect. Therefore, the method of adaptive signal decomposition and SVM is introduced into the signal preprocessing link, and the corresponding recognition process is established. In order to improve the performance of the support vector machine, the article uses measurement learning method to obtain the measurement learning and uses the measurement learning to replace the Euclidean distance of the Gaussian kernel function of the support vector machine. The SVM method of adaptive signal decomposition and the SVM method of principal component analysis are introduced into the preprocessing process of the note signal, and then the preprocessed signal is reconstructed in phase space, and the corresponding recognition process is established. The method of directly reconstructing the phase space of the original signal has higher accuracy and can be applied to the note recognition of continuous music segments. The final experimental results show that, compared with the current popular piano score recognition algorithm, the recognition accuracy of the proposed piano score recognition algorithm is improved by 3.5% to 12.2%.

## 1. Introduction

With the development of digital information technology in the 21st century, many applications based on music signal analysis, such as automatic labeling of music, music score translation, and music retrieval, have higher requirements for analysis results [1]. However, due to the complex composition of music signals, even for fully digitized signals, there is still no more complete method to analyze them in detail [2]. Piano score recognition is one of the important research issues in music signal processing. It plays an important role in song cover recognition, audio matching, and music recommendation systems [3]. From a signal perspective, we are concerned about two characteristics of audio: time and frequency. Most of the audio signal processing is also focused on the time-frequency analysis of music and frequency images and various statistical methods cannot achieve a good trade-off between time and frequency, so that audio processing has not been greatly improved [4]. The design of piano score notes feature and the selection of measurement learning models have always been the most active research content in the field of piano score note recognition. The content of piano music notes is not only an expression of the creator's emotions, but also an external representation of the music spectrum structure [5]. Therefore, the recognition of musical piano notes is inseparable from the knowledge of various aspects such as signal processing. According to the different processing domains, the single-tone estimation method can be divided into four categories: time domain method, frequency domain method, time-frequency domain method, and cepstral domain method [6]. Among them, the short-time autocorrelation method, the harmonic peak method, the wavelet analysis method, and the cepstrum method have outstanding detection effects in each category. However, occasionally there will be situations where higher harmonic components are greater than the fundamental frequency components in music signals, which will make the detection error of the harmonic peak method [7].

The article "Recognition of Continuous Music Segments Based on the Phase Space Reconstruction Method" was retracted in 2023. Reasons: unreliable results or conclusions; concerns about the data; concerns about the peer review; concerns about the citations.

Liu et al. [8] first compressed the signal spectrum energy to 12 musical scales based on music harmonic information and music theory knowledge and proposed to use 12-dimensional Pitch Class Profile (PCP) as the note feature of piano music scores. The piano score notes of the music are transcribed. Corpuz [9] proposed the Harmonic Pitch Class Profile (HPCP) feature and used it in the piano score recognition system. The experimental results show that the HPCP feature can effectively reduce the influence of the type of instrument on the notes of the piano score. Mello et al. [10] use the Enhanced Pitch Class Profile (EPCP) feature combined with the harmonic product spectrum and the PCP feature. EPCP superimposes and maps the harmonic energy by multiplication instead of summation, so that the distinction between simple chords is more obvious, and the effect of relatively complex piano notation patterns is poor, so it is rarely used. In addition to that, in recent years, scholars have further introduced ideas such as matrix analysis into the design of musical notes in piano scores. For example, Sun et al. [11] proposed a new type of NNLS-PCP feature based on Non-Negative Least Square (NNLS) solution. Before mapping the spectrum to the PCP vector, this feature obtains the frequency values corresponding to 84 notes through a priori knowledge and generates the dictionary based on this. Each element in the dictionary represents the fundamental frequency and its harmonic frequency corresponding to a note. Then they used the approximate *x* of the obtained spectrum and performed the mapping between the approximate spectrum and the PCP feature [12]. Through prior knowledge, this method can effectively solve the crosstalk of the fundamental frequency and harmonic frequency of the note during the mapping [13]. In order to enhance the robustness of the PCP feature to the notes of piano scores played by different timbre instruments, Liang et al. [14], based on the discrete cosine transform and the Mel frequency, proposed a Mel logarithmic PCP feature. A more practical type of multitone estimation method is the cyclic extraction method, which was first proposed by Patel and Chauhan [15]. Its idea is to regard the multitone signal as the superposition of multiple single-tone signals and then use a two-step loop to perform one by one estimate. In theory, it can deal with a mixture of countless single tones, and the detection result is particularly good for a mixture composed of random frequencies. But for music signals, the detection results are not satisfactory [16, 17]. In response to the existing problems, Noroozi et al. [18] also proposed an improved loop extraction method based on the principle of spectral smoothing. In this way, it is possible to avoid other harmonics that repeat the fundamental frequency and the detected fundamental frequency from being removed from the signal after the current detection, which will affect the next detection. However, there is no universal standard for the principle of spectral smoothing, which reduces its applicability [19–21].

The article "Recognition of Continuous Music Segments Based on the Phase Space Reconstruction Method" was retracted in 2023. Reasons: unreliable results or conclusions; concerns about the data; concerns about the peer review; concerns about the citations.

This article uses the method of measurement learning, according to the characteristics of the notes of the piano score, with supervised learning from the prior knowledge of the question itself to a measurement learning measurement matrix. Through this distance measurement, the original feature space is projected to a space with higher class discrimination, so that, in the projected feature space, the distribution of feature vectors with the same label is more compact, and the interval between feature vectors with different labels is larger. We further use measure learning to improve the Euclidean distance in the original SVM Gaussian kernel function, so that the improved measure learning-based SVM has better category discrimination. This article focuses on the aspect of frequency and on the basis of obtaining its accurate information, to the greatest extent to approximate the original signal. Through the processing of the approximation signal, the purpose of analyzing the original signal is achieved, and combined with the statistical measurement learning method, the single-tone signal is recognized. By collecting audio information from a single frequency level to obtain an accurate approximation of the signal, the approximation format is unified, the complex time-frequency analysis is transformed into a signal to matrix transformation, and the approximation format is detected with the measurement learning method, which improves the adaptability.

## 2. Construction of Piano Music Note Recognition Algorithm Model Based on Measure Learning Support Vector Machine

### 2.1. Support Vector Machine Hierarchical Spatial Distribution

Support Vector Machine (SVM) is a maximum boundary classifier, which has good robustness to outliers. SVM maps the feature vectors one by one into labeled outputs through strict mapping relationships. SVM is established on the basis of the dimension theory and the principle of structural risk minimization in the statistical learning theory. It is based on the limited sample information (training sample) in the model complexity and the learning ability to find the best compromise, so that it has the best generalization ability [22–24].  Figure 1 shows the hierarchical spatial distribution of support vector machines.

The key step of feature acquisition is to model the harmonic components corresponding to the piano score notes in the music signal spectrum and the nonharmonic components corresponding to the sparse and large noises and to obtain an optimization problem through augmented Lagrangian multiplication. The submethod is used to solve the problem, and finally the characteristic with better performance is obtained. This feature can remove large and sparse noise in the signal and reconstruct the harmonic information in the music signal, so that the feature contains more stable and pure harmonic information [25–27].

(1) $$\begin{array}{c} X\left[t|x\left(t\right)\right]=\left\{t\in R|x\left(1\right),x\left(2\right),\ldots ,x\left(t\right)\right\},\\ y\left(n\right)=A\times X\left(n\right)-t\times x\left(n-1\right). \end{array}$$

The signal preprocessing uses the empirical mode decomposition method. SVM is a smoothing process for a signal, and the result is to decompose the fluctuation or trend of different scales in the signal to produce a series of data series with different characteristic scales. Each series is called an intrinsic mode function.

(2) $$\begin{array}{c} h\left(x\right)=\left\{\begin{array}{cc} \varepsilon \left(i,n\right)\times x\left(t\right), & 0<t<1,\\ \delta \left(i,n\right)\times x\left(t\right), & t>1,\\ y\left(n\right)\times x\left(t\right), & t<0. \end{array}\right. \end{array}$$

After adding the signal preprocessing link, it is necessary to determine the number of characteristic subsignals after decomposition and determine the optimal phase space reconstruction parameters corresponding to each characteristic subsignal. When the cumulative contribution rate of the current *k*-level principal components reaches 85%, it indicates that the previous *k*-level principal components basically contain all the information contained in the test data.

(3) $$\begin{array}{c} f\left(x+1\right)-f\left(x\right)=\partial \frac{y\left(x,n\right)}{{\left\|d\left(n\right)\right\|}^{2}}d\left(n\right). \end{array}$$

In addition, because the feature vectors corresponding to some piano score types have a certain degree of similarity, the feature vectors corresponding to different piano score notes are likely to have a small Euclidean distance, which makes the classification accuracy of the support vector machine not high.

(4) $$\begin{array}{c} \bar{x^{2}}\left(k,n\right)-{\left|x\left(k,n\right)\right|}^{2}-2\left|\bar{x\left(k,n\right)}\right|\times \;\cos\;\alpha =0. \end{array}$$

We hope that the classification process is a process of measurement learning. In fact, there are many classifiers that meet the above requirements, and what we are looking for is an optimal classifier that satisfies the maximum separation of data points belonging to two different classes, so this hyperplane is called the maximum separation hyperplane.

(5) $$\begin{array}{c} \left\{\begin{array}{c} \frac{\alpha \left(x\right)-\alpha \left(x-1\right)}{2\pi x}=1,\\ \frac{\beta \left(x\right)-\beta \left(x-1\right)}{2\pi x}=1. \end{array}\right. \end{array}$$

For a musical instrument, the sound it plays is of course caused by its vibration, but the strength and duration of the frequency vibration that constitutes the note must be measured by the amplitude.

(6) $$\begin{array}{c} g\left(x,k\right)=\frac{1}{n}\times \sum_{i=1}^{n}\left(1-\alpha \left(x\right)\right)\times \left(1-\beta \left(x\right)\right)\times x\left(t\right). \end{array}$$

The article "Recognition of Continuous Music Segments Based on the Phase Space Reconstruction Method" was retracted in 2023. Reasons: unreliable results or conclusions; concerns about the data; concerns about the peer review; concerns about the citations.

### 2.2. Measure Learning Recognition Algorithm

In general, the adaptive signal decomposition of the music signal using the empirical mode decomposition method will generate a large number of subsignals, and most of the subsignals contain relatively little information. If all are determined as features in the case of subsignals, it will greatly increase the time required for the construction and recognition of the classifier and reduce the efficiency. Therefore, it is necessary to determine the signal containing more information as the characteristic subsignal from the decomposed subsignals.

(7) $$\begin{array}{c} W\left(x\right)=\left[\begin{array}{cccc} \frac{x\left(1\right)}{g\left(k,1\right)} & \frac{x\left(2\right)}{g\left(k,2\right)} & ... & \frac{x\left(n\right)}{g\left(k,n\right)}\\ 1 & 0 & ... & 0\\ 0 & 1 & ... & 0\\ 0 & 0 & ... & 1 \end{array}\right]. \end{array}$$

By observing the decomposed subsignal image and its corresponding spectrum image, it can be found that the first two subsignals after decomposition contain more information. Therefore, the first two subsignals after decomposition are determined as characteristic subsignals. After determining the number of characteristic subsignals, it is also necessary to determine the delay time and embedding dimension corresponding to each characteristic subsignal during phase space reconstruction.

Therefore, we cannot measure the gap between the selected hypothetical model and the real model. The spectrum before compression is called the original spectrum; then the compressed spectrum is compared with the original spectrum. For example, if the sampling coefficient is set to 2, then the first vertex in the original spectrum corresponds to the second vertex in the compressed spectrum. It corresponds to the third vertex in the compressed spectrum; when the original frequency spectrum and all compressed frequency spectrums are correspondingly multiplied, the result can clearly show the position of the fundamental frequency.

Figure 2 shows a schematic diagram of the measure learning recognition algorithm. After obtaining a classifier, we can approximate the error with the real model with certain quantities we have already mastered. The most intuitive method is to use sample data to classify the sample data with the obtained classifier and compare the result with the real classification result (still sample data). The difference between them is called the empirical risk. Algorithmically, the real number frame is used in the approximation process to avoid the solution of the high-order band matrix. The recognition process uses the normalized vector principle to standardize the amplitude range, so that the features at any time have a standard representation, which is more conducive to training and recognition. Theoretically speaking, an audio signal generated by a monophonic melody, the amplitude matrix A, obtained after the frame is approximated, each row of which should contain only the amplitude of one note, that is, the basis of the note.

The article "Recognition of Continuous Music Segments Based on the Phase Space Reconstruction Method" was retracted in 2023. Reasons: unreliable results or conclusions; concerns about the data; concerns about the peer review; concerns about the citations.

Table 1 shows the combination of musical note audio signal attributes. For a single-tone melody, it is composed of different notes, and after being played by a specific instrument, each note contains the unique overtone combination of this instrument, that is, the frequency combination. We can determine to construct the vector with the amplitude of the frequency as the feature and input it into the SVM as a training sample. From the knowledge of music theory, we also know that the different combinations of fundamental frequency and overtones are precisely the characteristics of the sound of the musical instrument, and it is the mark that distinguishes it from other musical instruments.

In theory, an audio signal is generated by a monophonic melody (only one note played at any time). Therefore, if we know the frequency composition of each note played by a certain musical instrument, then for the calculated row vector in A, the combination of its nonzero elements in turn corresponds to a note. After obtaining, we count the number of consecutive notes, so that the note and note duration of this audio signal can be obtained.

### 2.3. Weight Optimization of Piano Score Data

The method of principal component analysis SVM is a statistical method to reduce the dimensionality of the variable space. This method uses the orthogonal projection method to transform the original data from the high-dimensional variable space to the low-dimensional feature variable space, reducing the dimensionality of the variable space under the premise of the characteristic information, and the original data is retained. In this way, the analysis of the high-dimensional original data with the correlation between the variables is transformed into a low-dimensional space, thereby reducing the difficulty of analysis. In the case of unknown rules, an effective tool for classification is SVM.

Autocorrelation is effective for detecting repetitive patterns in a signal, such as detecting the period of a periodic signal covered by noise. In addition, the results of SVM analysis on other kinds of notes also show that the first four eigenvalues can represent the main components in the nonlinear matrix.  Figure 3 shows the comparison chart of the detection error broken lines of different groups of note data. It can be seen that, in the process of node length from 100 sampling points to 700 sampling points, the error ratio is also reduced from 3.6% to 1.5% in the worst case, but relative to the influence of low sampling times, the length of node is helpful to the accuracy of pitch detection and the accuracy of pitch extraction, but the effect is not as great as the impact of low sampling.

The article "Recognition of Continuous Music Segments Based on the Phase Space Reconstruction Method" was retracted in 2023. Reasons: unreliable results or conclusions; concerns about the data; concerns about the peer review; concerns about the citations.

Since the timbre characteristics of each instrument, that is, the composition of the frequency corresponding to the notes, are unknown, we need to build training data and input it into the SVM to build a classification model. First, the music signal is distributed to 9 nonoverlapping bands (nonoverlapping bands) through the filter group.  Figure 4 shows the feature vector processing process of musical note data information. In each frequency band, we use the autocorrelation algorithm to find the pitch of its corresponding frequency band. In the final stage, the pitches obtained in all frequency bands are fitted, and the desired pitch of the music is synthesized. Each row vector containing frequency and amplitude in A is exactly a feature vector containing audio information corresponding to the note, so it can be input into SVM for training.

For the traditional short-term analysis method, if the window width is 50 ms, taking the wav file with the highest sampling accuracy as an example, only 2205 samples can be obtained. Both accuracy and breadth are far from meeting the requirements of audio signal analysis. If the window width is increased to 1 s, the frequency domain resolution can reach the minimum difference 1 for distinguishing music signals. For a song with a tempo of 200, the 32th note lasts only 37.5 ms, which obviously cannot be detected. This is the bottleneck of traditional short-time analysis, which is a trade-off between the resolution of the time domain and the frequency domain. Because the music itself has signal stability in a short period of time, it exhibits a certain period, so the autocorrelation method can be used to detect the period of the music, and of course the fundamental frequency of the signal can be detected. We trade off model complexity and learning ability based on small sample data, hoping to achieve the best generalization ability measurement learning method. It can be found that the cumulative contribution rate of the first four eigenvalues can reach more than 90%.

## 3. Results and Analysis

### 3.1. Feature Extraction of Musical Notation Data

The masking of notes and missing notes during the performance of the music will have a certain impact on the recognition and transcription of the final piano score. Therefore, the extraction of robust PCP features is divided into two steps: reconstruction of the harmonic information in the signal spectrum and scale mapping. The frame method starts from the whole audio signal, first obtains accurate frequency information from a large window, and uses the known frequency to construct an approximation of the original signal. In this way, the main frequency information of the original signal is kept as close as possible to its time domain information, so as to achieve the analysis of the music signal.

The article "Recognition of Continuous Music Segments Based on the Phase Space Reconstruction Method" was retracted in 2023. Reasons: unreliable results or conclusions; concerns about the data; concerns about the peer review; concerns about the citations.

The two-tone connection recognition results of common piano notes are given; that is, the first note starts at 0 s, the second note starts at 0.5 s, and the number of recognition samples is 44100. From the data, it can be seen that, for the two-tone case, the classification is completely correct and does not include nonaudio internal notes; in most cases, the first note gets more recognition results, and the error is completely caused by this. This process is generally about 10–15 ms. Although theoretically speaking, the second note starts playing at 0.5 s, but its effective time will have a lag of 10–15 ms. That is to say, when the frequency contained in the second note is large enough to be classified, there is a 10–15 ms lag from the theoretical time.

Table 2 shows the statistical classification of the recognition results of piano score data. For the reliability and convenience of category labeling, the songs in the test music library and their corresponding labels are all from the music library on the Internet. We have selected a total of 480 songs in 6 categories. In this experiment, all music songs are in mp3 format, and their sampling rate is adjusted to 11025 Hz, and the bit rate is 16 kbps. It provides a software package for reading mp3 format music through MATLAB software. In this experiment, the length of 1024 is used for each frame. In the octave critical frequency band filter, because the sampling frequency of the test data is 11024 Hz, when it is decomposed into the critical frequency band, only the first 7 frequency bands are included in the effective frequency band, because the upper limit of the effective frequency is 5513 Hz. When calculating the 44th and 60th frames, the experimental data are as follows.

Each row of the amplitude matrix A obtained after the frame approximation should only contain the amplitude of one note. The usual method for detecting the starting point of a note is to find the “transient” area in the music signal; there are many definitions for the transient area, such as energy mutation points, short-term changes in the signal spectrum, etc. The above reduces the size of the data volume but refers to the audio signal as the input of a highly low sampling detection function and the role of the detection function to show the “instantaneous” in the original signal.

In this experiment, only the first 120 seconds of each song are intercepted for training or testing. Therefore, the time length of most songs is 3–5 minutes, so the first 120 seconds can already contain the basic characteristics of the song. For songs up to 120 seconds, a loop sampling method is adopted; that is, the beginning part of the song is connected to the end of the song.  Figure 5 shows the fan-shaped distribution diagram of the recognition accuracy of different sampling units. In the 120 seconds of each song, 2.6 seconds are used as a music segment; each music segment is further divided into smaller unit music frames. The sampling frequency occupied by each time period is 28.99%, 21.89%, 22.19%, 11.54%, and 15.38%, respectively. Each music segment is further divided into 64 music frames. Each music frame contains 512 sampling points, and adjacent frames overlap 64 sampling points.

The article "Recognition of Continuous Music Segments Based on the Phase Space Reconstruction Method" was retracted in 2023. Reasons: unreliable results or conclusions; concerns about the data; concerns about the peer review; concerns about the citations.

That is, the amplitude of the fundamental frequency and the overtone constituting the note and the amplitude of the frequencies contained in the notes that are not sounded at that moment are all zero. At the same time, due to the natural attenuation of audio, when the original feature data is processed by SVM, the projection feature of 95% of the original feature information is retained. After the SVM projection processing, the final feature of the dataset is reduced to 13 dimensions, and the feature of the dataset is reduced to 8 dimensions. Then, the SVM algorithm based on each kernel function is used to classify the data after SVM dimensionality reduction. It can be seen that after the original feature data is processed by SVM, the classification accuracy of each SVM is improved. This is because the original feature data after SVM projection and dimensionality reduction can effectively reduce aliasing and redundant information, thereby improving the accuracy of the final classification.

### 3.2. Simulation of Measure Learning Recognition Model

Firstly, the music fragment is sampled and processed with a sampling rate of 11025 Hz, and an audio signal with a length of node is generated. For the audio signal mode of this length, we use the window function *W* (*n*) to preprocess the audio signal, and the window shift length is 50% of the window width to obtain the windowed waiting. Then, we multiply the signal matrix by the Fourier transform matrix, the force is an *N* × *N* square matrix, and the rows of the matrix are the orthonormal basis, so that the frequency spectrum matrix of the framed signal is obtained as *M*. In the experiment, phase space reconstruction is performed on the original note signal, the first subsignal, and the second subsignal, the SVM principal component is extracted, and then the nonlinear feature construction is carried out. The piano score data set adopts MIDI format digital score files that contain piano score information such as pitch, beat, time, chord, speed, and channel.

The article "Recognition of Continuous Music Segments Based on the Phase Space Reconstruction Method" was retracted in 2023. Reasons: unreliable results or conclusions; concerns about the data; concerns about the peer review; concerns about the citations.

In order to obtain more features related to the difficulty of piano scores, this paper adopts the related features of difficulty as the feature space of this paper. Therefore, the feature space in this article includes all the difficulty and semantic features except the fingering complexity (which belongs to the information of the score labeling level, and MIDI scores does not contain this information), key signature (key signature is meta tag information); except for the fingering feature (also belongs to the label layer feature) all the features, a total of 22 features, form a 22-dimensional feature vector to represent the MIDI score. Given the recognition results of common triplet within 1 s, 50 samples are selected for recognition from the approximation data.  Figure 6 shows a matchstick graph of the attenuation rate of the note data signal based on measurement learning. From the figure, we can see that there are still notes that will get more detection results. This is caused by the crossover of notes, especially when the sound is not deliberately muted during performance, so that each note is naturally attenuated and played.

Either from the audio waveform graph or from the approximate amplitude graph, it can be clearly found that the previous note still has a strong amplitude at the note boundary. After normalization, the note with a weaker amplitude will be detected. However, although reducing the sampling rate increases the error percentage, the statistically obtained duration does not change much, and it has no effect on the translation of the score.

In the experiment, the 20 samples of each note signal were taken as test signals for the identification experiment.  Figure 7 shows the SVM-based note data recognition deviation box diagram. In addition, considering many situations in actual piano learning and teaching, music scores are divided into 4 difficulty levels, and a large number of music websites generally provide digital music scores with 4 difficulty levels (easy, beginning, intermediate, and advanced). The scalability of the algorithm in this paper is suitable for practical applications. We also collected 400 MIDI scores from the large music website to form a data set with 4 difficulty levels, each with 100 MIDI scores.

From the knowledge of music theory, we also know that the different combinations of fundamental frequency and overtones are precisely the characteristics of the sound of an instrument, and it is the mark that distinguishes it from other instruments. Among them, the delay time and embedding dimension of the original signal are determined as 5 and 9, the delay time and embedding dimension of the first subsignal are determined as 2 and 7, and the delay time and embedding dimension of the second subsignal are determined as 4 and 9. The nonlinear characteristics of the training signal are used for the construction of the SVM classifier, and the nonlinear characteristics of the test signal are used for the recognition experiment. According to the recognition results, after adding empirical mode decomposition and SVM preprocessing in the recognition process, the recognition accuracy rate is better than the method of directly using the phase space of the note signal to reconstruct the matrix, and the average accuracy rate is improved.

The article "Recognition of Continuous Music Segments Based on the Phase Space Reconstruction Method" was retracted in 2023. Reasons: unreliable results or conclusions; concerns about the data; concerns about the peer review; concerns about the citations.

### 3.3. Example Results and Analysis

The algorithms in this paper are all implemented with MATLAB software, and the computer environment used is a 32-bit Windows 7 operating system, with a built-in Intel I5-4200M processor and 4 GB of memory. In the experiment, in order to better evaluate the classification performance and generalization ability of the ML-SVM algorithm proposed in this paper, the ML-SVM algorithm is combined with logistic regression and linear kernel function in two musical score data sets of 9 and 4 difficulty. Each experiment was repeated 5 times independently, and a fivefold cross-validation was used, and the average accuracy rate was taken as the final recognition accuracy rate. At the same time, in order to evaluate the performance of the recognition algorithm more comprehensively, the 90% confidence interval of each algorithm result is also given.

Figure 8 shows the histogram comparison of the SNR (signal-to-noise ratio) of note data with the same algorithm. We use the B-spline frame twice to approximate the signal and the Gaussian frame to approximate the acoustic guitar *d* 1, and the error is measured. The characteristics of these three examples are clearly contrasted and can truly reflect the practical effects of the framework under various signal compositions. We see that, for signals with clear and clear frequencies, the result of frame approximation is very satisfactory.

In the actual playback of this signal, the error is very small, and human ears can hardly distinguish the difference. It can be seen that the error is larger at the beginning of the note and decreases with time. This is because plucked instruments are affected by factors such as plucking strength and angle, which will cause other strings at the beginning of the note. Resonance and the noise caused by flicking will therefore weaken over time.

Figure 9 shows the amplitude response curves of different note signal frequencies. In addition, when setting the music frequency, we only kept the 10 frequencies of the piano, with a maximum value of 1000 Hz. In actual recording, the effector will add harmony and simulation effects. These effects contain a lot of high-frequency signals, but these frequencies are discarded as noise. When the signal is actually played, the note restoration is highly recognizable, and the pitch and timbre information of the original signal is preserved, but it does not sound as bright and crisp as the original signal. This is precisely the result of discarding the high-frequency signal. We see that the response amplitude value is much lower than the previous two.

The article "Recognition of Continuous Music Segments Based on the Phase Space Reconstruction Method" was retracted in 2023. Reasons: unreliable results or conclusions; concerns about the data; concerns about the peer review; concerns about the citations.

Therefore, if we know the frequency composition of a certain musical instrument playing each note, then for the calculated row vector in A, the combination of its nonzero elements in turn corresponds to a note. This is caused by the upgrade of signal complexity. Due to the influence of the sound of the instrument itself, the superimposition of notes is serious, and it is also affected by the recording environment and the structure of the piano itself. Environmental noise and high-frequency overtones are more and more complicated than the previous two examples. In actual playback, the approach signal retains the main frequency composition of the original signal, the note recognition is high, the energy feedback is obvious, and the beginning and end of the note can be clearly heard. However, part of the timbre information is lost, and the recognition of the instrument is reduced. This is related to the piano's own frequency response range. The threshold of the main frequency selection can be lowered to improve the approximation effect.

In order to improve the generalization ability, we perform multiparameter approximation on the training audio and obtain different frequency combinations of the same note by adjusting the Fourier transform threshold and the frame translation distance. Numerical experiments show that SVM can recognize single-tone melody very well, and every moment is correctly classified into the frequency that appears in the audio, and no nonaudio frequency is recognized, so the recognition rate of the note is 100%. However, due to the attenuation nature of the audio signal and the setting of the playing time, in the intersecting zone the previous note is about to stop and the next note has been played.

Figure 10 shows the line comparison chart of the recognition accuracy of musical note signal algorithms. It can be seen that, in the two data sets, among several algorithms, the final recognition accuracy of the algorithm proposed in this paper is higher than that in [19], in [20], and in [21], especially in the data set. The proposed algorithm obtains a recognition accuracy rate of 90.67%, which is greatly improved compared to the 85.63% literature algorithm. And a narrower confidence interval indicates that the result is more stable and significant. Compared with theoretical expectations, when the sampling rate is 1000, the duration error is between 0.5% and 1.6%. If the sampling rate is reduced, not only can the classification accuracy be improved, but also the real-time processing requirements for music within 200 tempos can be met.

The article "Recognition of Continuous Music Segments Based on the Phase Space Reconstruction Method" was retracted in 2023. Reasons: unreliable results or conclusions; concerns about the data; concerns about the peer review; concerns about the citations.

## 4. Conclusion

The piano music note recognition system designed in this paper includes four main steps: audio input, spectrum preprocessing, feature calculation, and measurement learning support vector machine classification. Because the method of using fixed parameter values for different types of notes to extract the characteristic parameters will cause the loss of some nonlinear information of the notes and ultimately affect the recognition accuracy, this paper applies the method of adaptive signal decomposition to the signal preprocessing link. At the same time, in order to improve the recognition efficiency and reduce the time required for recognition, the paper also uses the SVM method to extract the principal components of the nonlinear features for the construction of the classifier and specific note recognition experiments. Then we propose a new method of monophonic melody recognition based on frame approximation theory by using the accurate characteristics of the Fourier transform in the frequency domain, the frequency of energy concentration is detected in a large window, and then the idea of least squares is used to approximate the original signal, and on the basis of preserving the time-frequency characteristics of the original signal to the greatest extent, the audio is standardized and organized. Combining support vector machines based on statistical methods to recognize notes, it has the characteristics of supporting multiple frequencies and multiple notes, fast recognition, expandable models, and strong generalization capabilities. Among them, the spectrum preprocessing mainly uses the nuclear norm convex optimization technology to reconstruct the harmonic components in the original audio and adds a norm penalty term to enhance the robustness of the calculated spectrum against sparse noise; then the scale mapping is used to extract the features of harmonic information, and finally we input these features into the support vector machine based on measurement learning.

## Figures and Tables

**Figure 1:** Hierarchical spatial distribution of support vector machines.

**Figure 2:** Schematic diagram of measure learning recognition algorithm.

The article "Recognition of Continuous Music Segments Based on the Phase Space Reconstruction Method" was retracted in 2023. Reasons: unreliable results or conclusions; concerns about the data; concerns about the peer review; concerns about the citations.

**Figure 3:** Comparison of broken lines of detection error for different groups of note data.

**Figure 4:** Feature vector processing process of musical note data information.

**Figure 5:** Fan-shaped distribution diagram of recognition accuracy of different sampling units.

**Figure 6:** Match stick graph of attenuation rate of note data signal based on measurement learning.

**Figure 7:** Box diagram of note data recognition deviation based on SVM.

**Figure 8:** The comparison chart of SNR of note data of different algorithms.

**Figure 9:** Amplitude response curves of different note signal frequencies.

**Figure 10:** The comparison chart of the broken line of the recognition accuracy of the musical note signal algorithm.

**Table 1:** Musical note audio signal attribute combination.

Node serial	Frequency (Hz)	Duration ratio (%)	Standard deviation
1	2000	87	1.81
2	4000	91	0.98
3	6000	79	2.02
4	8000	56	1.96
5	10000	54	0.59
6	12000	69	0.64
7	14000	88	0.77

**Table 2:** Statistical classification of piano score data recognition results.

Node number	Frame number	Resolution (Hz)	Time delay (ms)	Error (%)
1	10	3.60	15	3.10
2	20	3.50	17	2.70
3	30	2.90	18	3.30
4	40	2.70	16	3.10
5	50	3.10	19	2.90

## Data Availability

The data used to support the findings of this study are available from the corresponding author upon request.

## References

[1] Mitiche I., Morison G., Nesbitt A., Hughes-Narborough M., Stewart B. G., Boreham P. (2018). Classification of EMI discharge sources using time-frequency features and multi-class support vector machine. *Electric Power Systems Research*.

[2] Adil Abboud S., Al-Wais S., Abdullah S. H. (2019). Label self-advised support vector machine (lsa-svm)—automated classification of foot drop rehabilitation case study. *Biosensors*.

[3] Sevakula R. K., Verma N. K. (2017). Compounding general purpose membership functions for fuzzy support vector machine under noisy environment. *IEEE Transactions on Fuzzy Systems*.

[4] Wu C. T., Dillon D. G., Hsu H. C. (2018). Depression detection using relative EEG power induced by emotionally positive images and a conformal kernel support vector machine. *Applied Sciences*.

[5] Chahine K. (2018). Rotor fault diagnosis in induction motors by the matrix pencil method and support vector machine. *International Transactions on Electrical Energy Systems*.

[6] Azad-Manjiri M., Amiri A., Saleh Sedghpour A. (2020). ML-SLSTSVM: a new structural least square twin support vector machine for multi-label learning. *Pattern Analysis and Applications*.

[7] Ardianto R., Rivanie T., Alkhalifi Y., Nugraha F. S., Gata W. (2020). Sentiment analysis on E-sports for education curriculum using naive bayes and support vector machine. *Jurnal Ilmu Komputer dan Informasi*.

The article "Recognition of Continuous Music Segments Based on the Phase Space Reconstruction Method" was retracted in 2023. Reasons: unreliable results or conclusions; concerns about the data; concerns about the peer review; concerns about the citations.

[8] Liu W., Zhang L., Tao D., Cheng J. (2017). Support vector machine active learning by hessian regularization. *Journal of Visual Communication and Image Representation*.

[9] Corpuz R. S. A. (2021). Categorizing natural language-based customer satisfaction: an implementation method using support vector machine and long short-term memory neural network. *International Journal of Integrated Engineering*.

[10] Mello A. R., Stemmer M. R., Koerich A. L. (2020). Incremental and decremental fuzzy bounded twin support vector machine. *Information Sciences*.

[11] Sun Z., Guo Z., Liu C., Wang X., Liu J., Liu S. (2017). Fast extended one-versus-rest multi-label support vector machine using approximate extreme points. *IEEE Access*.

[12] Wang X., Yang Y., Xu Y. (2020). Predicting hypoglycemic drugs of type 2 diabetes based on weighted rank support vector machine. *Knowledge-Based Systems*.

[13] Rizwan A., Iqbal N., Ahmad R., Kim D.-H. (2021). WR-SVM model based on the margin radius approach for solving the minimum enclosing ball problem in support vector machine classification. *Applied Sciences*.

[14] Liang B., Fazekas G., Sandler M. (2018). Measurement, recognition, and visualization of piano pedaling gestures and techniques. *Journal of the Audio Engineering Society*.

[15] Patel E., Chauhan S. (2017). Raag detection in music using supervised machine learning approach. *International Journal of Advanced Technology and Engineering Exploration*.

[16] Singh P., Bachhav D., Joshi O. (2019). Implementing musical instrument recognition using cnn and svm. *International Research Journal of Engineering and Technology*.

[17] Ahmad S., Agrawal S., Joshi S. (2020). Environmental sound classification using optimum allocation sampling based empirical mode decomposition. *Physica A: Statistical Mechanics and Its Applications*.

[18] Noroozi F., Kaminska D., Sapinski T. (2017). Supervised vocal-based emotion recognition using multiclass support vector machine, random forests, and adaboost. *Journal of the Audio Engineering Society*.

[19] Cheng C.-F., Rashidi A., Davenport M. A., Anderson D. V. (2017). Activity analysis of construction equipment using audio signals and support vector machines. *Automation in Construction*.

[20] Othman A., Direkoğlu C. (2020). Recognizing musical notation using convolutional neural networks. *Avrupa Bilim ve Teknoloji Dergisi*.

[21] Seo Y.-S., Huh J.-H. (2019). Automatic emotion-based music classification for supporting intelligent IoT applications. *Electronics*.

[22] Sadewo W., Rustam Z., Hamidah H., Chusmarsyah A. R. (2020). Pancreatic cancer early detection using twin support vector machine based on kernel. *Symmetry*.

The article "Recognition of Continuous Music Segments Based on the Phase Space Reconstruction Method" was retracted in 2023. Reasons: unreliable results or conclusions; concerns about the data; concerns about the peer review; concerns about the citations.

[23] Schleif F.-M., Tino P. (2017). Indefinite core vector machine. *Pattern Recognition*.

[24] Verde L., De Pietro G., Sannino G. (2018). Voice disorder identification by using machine learning techniques. *IEEE Access*.

[25] Chen Y., Wu W., Zhao Q. (2019). A bat-optimized one-class support vector machine for mineral prospectivity mapping. *Minerals*.

[26] Birajdar G. K., Patil M. D. (2020). Speech/music classification using visual and spectral chromagram features. *Journal of Ambient Intelligence and Humanized Computing*.

[27] Dias Canedo E., Cordeiro Mendes B. (2020). Software requirements classification using machine learning algorithms. *Entropy*.

